The article "Segmentation and Classification of Encephalon Tumor by Applying Improved Fast and Robust FCM Algorithm with PSO-Based ELM Technique" was published in 2022. Journal: Comput Intell Neurosci.

# Segmentation and Classification of Encephalon Tumor by Applying Improved Fast and Robust FCM Algorithm with PSO-Based ELM Technique

**DOI:** 10.1155/2022/2664901

**Published:** 2022-07-31

**Authors:** Srikanta Kumar Mohapatra, Premananda Sahu, Jasem Almotiri, Roobaea Alroobaea, Saeed Rubaiee, Abdullah Bin Mahfouz, A. P. Senthilkumar

**Affiliations:** ^1^Chitkara University Institute of Engineering and Technology, Chitkara University, Rajpura, Punjab, India; ^2^SRM Institute of Science and Technology, Ghaziabad, UP, India; ^3^Department of Computer Science, College of Computers and Information Technology, Taif University, Taif 21974, Saudi Arabia; ^4^Department of Industrial and Systems Engineering, College of Engineering, University of Jeddah, Jeddah, Saudi Arabia; ^5^Department of Chemical Engineering, University of Jeddah, P.O. Box 80327, Jeddah 21589, Saudi Arabia; ^6^Jigjiga University, Somali Regional State, East Africa, Jijiga, Ethiopia

## Abstract

Nowadays, so many people are living in world. If so many people are living, then the diseases are also increasing day by day due to adulterated and chemical content food. The people may suffer either from a small disease such as cold and cough or from a big disease such as cancer. In this work, we have discussed on the encephalon tumor or cancer which is a big problem nowadays. If we will consider about the whole world, then there are deficiency of clinical experts or doctors as compared to the encephalon tumor affected person. So, here, we have used an automatic classification of tumor by the help of particle swarm optimization (PSO)-based extreme learning machine (ELM) technique with the segmentation process by the help of improved fast and robust fuzzy C mean (IFRFCM) algorithm and most commonly feature reduction method used gray level co-occurrence matrix (GLCM) that may helpful to the clinical experts. Here, we have used the BraTs (“Multimodal Brain Tumor Segmentation Challenge 2020”) dataset for both the training and testing purpose. It has been monitored that our system has given better classification accuracy as an approximation of 99.47% which can be observed as a good outcome.

## 1. Introduction

Whenever we are going to do some investigation work, then first of all, we have to find out actually what is our motive. Here, our basic motivation is from magnetic resonance image (MRI), the pictures will segment first, the features or characteristics will remove, and finally that will be categorized whether it is cancerous or noncancerous.

To carry out the above issue, we have to use or apply some technique or tool which can all be corelated to each other. Initially, if we will discuss about the magnetic resonance image, then it is a leading technique to scan the whole brain and monitor the disease such as tumor. As our study is related to the neural network, it will explore the pictures and integrate them into 3-dimensional which can be used for better forecasting [1]. Next, the above processes have been used to help the clinical experts for detection of cancerous encephalon tumor in an effective manner. One more thing to be discussed here is that if the encephalon tumor spread steadily, some irregular activities have shown to the patients such as “vision problem and vomiting” which can cause a great problem if early investigation has not taken by the clinical experts [2]. If the physical examination has carried out from MRI, then it may be very heavy or time taking task for the clinical practitioners due to composite shape of cancer area as well as some dotted spots inside the MRI picture. In this paper, some systematic work has been conducted that can determine that this is fully automatic and it may help the clinical experts. Initially, when somebody feels like drowsiness [3], memory problems, and some severe headache problem, there may be a chance for growing a tumor inside the brain [4–6]. So, that particular person has to visit the nearest hospital for scanning the brain. Regarding the scanning process, MRI is the best method to find out the clear picture of the brain as well as it has been built by some advance technologies [7]. For better understanding of MRI, we can use functional MRI due to the different types of activities that can be detected by changing with the blood vessels [8, 9]. After scanning, it needs to divide the pictures as some dotted or some odd pictures will present. For segmentation purpose, we have used the improved fast and robust fuzzy C mean technique as it can remove the noisy images [10]. After segmentation, some characteristics or features have to be removed from the input data so that the precision may be improved. For this purpose, we have used the frequently used technique gray level co-occurrence matrix. After removing some attributes, they will be nutrified as input to the particle swarm optimization based extreme learning machine for the categorization point of view which can be further divided into cancerous or noncancerous cells. This technique has been utilized to maximize the input and hidden layers that can be computed for tumor classification [11] as well as the bias along with weights. After successfully applied all the above techniques, it is the time for implementation process. Regarding this, we have used BraTs (“Brain Tumor Segmentation Challenges”) for both the training as well as testing purpose.

The rest of this investigation work has been formulated in the following manner: Section 2 describes related work, Section 3 describes methodology, Section 4 describes result and discussion, and Section 5 describes conclusion followed by future work.

## 2. Related Work

Here, the authors mainly focused into segmentation and feature removal followed by categorization. Previously, some authors have worked in the above processes and we are going to discuss some of them as follows:

The authors in [12] have developed a compound forecasting model for perception and segmentation of brain tumor. In this work, they have used the hierarchical K-means clustering method with super rule tree for the above prediction process. Here, the FCM method has been used for the segmentation method which gives as an approximation of 88.9% of accuracy as well as they have concluded that their model can be used for multifaceted resection process also. Hua et al. [13] proposed the image segmentation method by a novel approach such as the improved multiview FCM clustering method. In their investigation work, they have also compared with the several clustering algorithms and their proposed model gives best accuracy. For implementation purpose, they have used the Simulated Brain Database but for the high-dimensional multiview function, their proposed model may give some less accuracy. Hu et al. [14] has been investigated the encephalon disease forecasting process by the help of fuzzy system. Here, they have forecasted the image segregation regarding encephalon tumor process by “Hybrid Pyramid U-Net” model. They have also compared their proposed model with “local density clustering FCM and adaptive FCM” for their experimental purpose. Their model has given better classification accuracy but for the shape and texture characteristics, it has given some less accuracy.

Kumar et al. [11] has been proposed an automatic forecasting model for encephalon tumor identification and categorization. Here, they have examined a lot of things regarding the above process, but our main intention in this survey is to only the feature extraction process. In this work, they have used the mostly common method, gray level co-occurrence matrix, for feature reduction and it gives an awesome performance. They have again suggested that if some texture and shape features can be used in addition to GLCM, and then it may give best accuracy. Sathi and Islam [15] classified the encephalon tumor by ANN and extracted the features by some hybrid methods such as “Gabor filter and discrete wavelet based as well as GLCM” where they have used 6 characteristics by which the features has been extracted. Again, they have indicated that after the features have been extracted, it has given an awesome performance to detect the brain tumor. Mall et al. [16] extracted all the features from an X-ray image. Here, they have also used the GLCM technique for the above purpose. In their work, they have classified bone fracture instead of encephalon tumor detection. They have used 12 characteristics for the extraction purpose and have noticed a good result.

Velmurugan and Velmurugan [17] proposed the encephalon tumor classification process by the particle swarm intelligence method. By their investigation method, axial as well as coronal plane also detected. Their model has also given better accuracy rate, and some more machine learning approaches can be used for sagittal plane which can dissociate into sections from the left and right side of encephalon then it may give more accuracy rate. Khan et al. [18] has classified the encephalon cancer process by the extreme learning method with the association of correntropy via the mutual learning process. In their work, they have also used the BraTs dataset for experimental purpose and their outcomes are immovable. Ayane et al. [19] proposed the classification of encephalon tumor by the PSO-ELM technique and executed across the embedded system. They have used here the dataset “Harvard Medical School” for both the training as well as testing purpose. According to the researchers, their work has produced great achievement for finding the outcome and it may be helpful to the clinical experts for classifying the encephalon tumor as cancerous or noncancerous [20, 21].

From the above survey, it has been observed that for detection and classification of encephalon tumor not only the feature removal or classification are required but also some extra attributes such as texture characteristics and coronal as well as sagittal suture are also used which we are going to implement in our work.

## 3. Methodology

In this work, mainly the researchers have focused into noncancerous tissues which may be found from segmentation [22] as well as the feature reduction method via magnetic resonance image [23]. This investigation work has flaunted in Figure 1.

This above diagram has been expanded through the following steps:

- Initially, the image has possessed by MRI [24].
- Then, this image has been segmented by our IFRFCM technique [25].
- Next, some features have removed by the most common method GLCM. [26].
- After successful removal of features, the data then processed and proceeded for validation.
- The next process is classification which can be estimated by PSO-ELM. [27].
- Finally, the tumor has been detected as cancerous or noncancerous.

### 3.1. Proposed IFRFCM for Image Segmentation

If the tumor is going to be detected from MRI, some noise has to be removed from those images. As described by the author [2], the above technique has the ability to remove the noise. As this technique supports “Wiener Filter” that has the ability to observe the noisy images, here the objective function must be required. Now, the objective function as per FCM is [28, 29]

(1) $$\begin{array}{c} J_{0}=\overset{N}{\underset{p=1}{\sum }}\overset{C}{\underset{q=1}{\sum }}\sigma_{qp}^{v}x_{p}-p_{q}^{2}+\overset{N}{\underset{p=1}{\sum }}\overset{C}{\underset{q=1}{\sum }}G_{pq}, \end{array}$$

where *G*_*pq*_ = fuzzy factor and it is defined as

(2) $$\begin{array}{c} G_{pq}=\underset{\begin{array}{c} r\in N_{p}\\ p!=r \end{array}}{\sum }\frac{1}{d_{pr}+1}{\left(1-\sigma_{qr}\right)}^{v}x_{r}-p_{q}^{2}, \end{array}$$

where

 
*x*_*p*_, *x*_*r*_ = pixels
 
*d*_*pr*_ = spatial Euclidian distance between *x*_*p*_ and *x*_*r*_
 
*N*_*p*_ = set of neighbors
 
*σ*_*qp*_ = Fuzzy membership of *p*th pixel with respect to *q*
 
*σ*_*qr*_ = neighbor of *σ*_*qp*_
 
*N* = total number of pixels in image
 
*C* = cluster centre
 
*V* = fuzziness of significant division

With the diminish of analytical intricacy, the fuzzy division matrix is defined as

(3) $$\begin{array}{c} G_{pq}^{\prime }=\underset{\begin{array}{c} r\in N_{p}\\ p!=r \end{array}}{\sum }\frac{\log{\left(\mu \right)}^{\alpha }}{\text{exp}\left(d_{pr}\right)+1}{\left(\sigma_{qr}\right)}^{v}x_{r}-p_{q}^{2}, \end{array}$$

where

 
*μ* = gray value of image
 
*α* = precision variable between 0 and 1

As we have to extract the marked objects from image, so some additional operations such as dilation and erosion are required which belongs to morphological reconstruction. Now, this type of image is indicated as *γ*_*z*_and it is described as [30–32].

(4) $$\begin{array}{c} \gamma_{z\;}=\;R_{d}^{c}\;\left(f\right), \end{array}$$

where

 
*R*_*d*_^*c*^ = morphological closing reconstruction
 
*f* = original image

Now, by the help of morphological closing reconstruction, the above objective function may be adjusted as

(5) $$\begin{array}{c} J_{0}=\overset{C}{\underset{q=1}{\sum }}\overset{h}{\underset{z=1}{\sum }}\left[\sigma_{qz}^{v}\gamma_{z}-p_{q}^{2}\right]+\overset{C}{\underset{q=1}{\sum }}\overset{h}{\underset{z=1}{\sum }}G_{qz}, \end{array}$$

where *σ*_*qz*_ = degree of membership of gray value *z* in cluster *q*

Now, here, the fuzzy factor may be adjusted as

(6) $$\begin{array}{c} G_{qz}^{\prime }=\underset{\begin{array}{c} r\in h_{p}\\ p!=r \end{array}}{\sum }\frac{\log{\left(\mu \right)}^{\alpha }}{\text{exp}\left(d_{pr}\right)+1}{\left(\sigma_{qr}\right)}^{v}\gamma_{z}-p_{q}^{2}. \end{array}$$

Now, the membership partition matrix appeared as *S* and it can be described as

(7) $$\begin{array}{c} S=\;{\left[\sigma_{qr}\right]}^{c*h}. \end{array}$$

As we have discussed above, the Wiener Filter has the ability to observe the noisy image [20], so the new membership partition matrix *S*′ can be described as

(8) $$\begin{array}{c} S{}^{\prime }=\text{Wiener}\left[S\right]. \end{array}$$

### 3.2. Proposed GLCM Technique for Feature Removal

As MRI consists of so many pictures that has to be captured, so for reduction of large number of pictures to the noisy picture, there is a removal technique is used [33, 34]. This is called as feature extraction process [35]. In this work, we have used the GLCM technique for feature extraction where it collects superior stage of facts of a picture such as structure, size, and color etcetera [36].

The previous researchers have used either only the GLCM technique or at max one of the feature like text characteristics or coronal or sagittal suture may be used [37]. However, here we have used all the above three features have been used for feature removal. All the process has described below:

- In texture features, initially, by the help of image processing technique, the images are combined to find the best outcome. Finally, the GLCM technique calculates the gray image and some texture features have been removed [38].
- In coronal plane, the MRI images have been divided into front and back where the images are clearly visible and easy for removal [39].
- In sagittal suture, the MRI images have divided into left from right so that the actual contusions are clearly visible [40].

From the above processes, it comes to know that GLCM with some characteristics have the ability to remove the features.

### 3.3. Proposed PSO-ELM Technique for Image Classification

Here, we have used one of the new techniques for classifying the tumor as cancerous or noncancerous, i.e., PSO-ELM. As PSO is an optimization technique, it has the ability to optimize the ELM parameters like weight and bias as well as the hidden neurons. From those hidden neurons, the above technique can find the good accuracy [41]. Here, the automatic categorization of encephalon tumor accomplished through our suggested PSO-ELM model [42]. Here, the weights are updated by the PSO technique [43] for finding each particle's best position by calculating the mean, so that it can upgrade to high competence.

It is a very useful as well as proficient training algorithm. Now, the output of ELM, *Y*, is determined as

(9) $$\begin{array}{c} Y=\overset{H}{\underset{i=1}{\sum }}v_{i}b_{i}\left(x\right)=\overset{H}{\underset{i=1}{\sum }}v_{i}b\left(w_{i}\times x_{J}+k_{i}\right),\;J=1,\;2,\;3,\ldots ,\;N, \end{array}$$

where *H* = number of hidden units, *N* = number of training samples, *w* = weight vector between input and hidden layer, *v* = weight vector between hidden and output layer, *b* = activation function, *k* = bias vector, and *x* = input vector.

Now, if we will assume beta matrix as special matrix, the output *Y* will be considered as

(10) $$\begin{array}{c} Y=Z*\beta , \end{array}$$

where *z* = hidden layer output matrix and it can be described as

(11) $$\begin{array}{c} Z={\left[\begin{array}{c} b\left(w_{1}\times x_{1}+k_{1}\right)\;\ldots \\ \vdots \\ b\left(w_{1}\times x_{1}+k_{1}\right)\;\ldots \\ b\left(w_{H}\times x_{1}+k_{H}\right)\\ \vdots \\ b\left(w_{H}\times x_{N}+k_{H}\right) \end{array}\right]}_{N\times H}. \end{array}$$

Now, equation (11) is a linear system which may be solved by

(12) $$\begin{array}{c} \beta =z†d, \end{array}$$

where *z*† = Moore-Penrose Generalized Inverse of Matrix *z* and

(13) $$\begin{array}{c} \beta =\left[\begin{array}{c} \begin{array}{c} \beta_{1}\\ \beta_{2}\\ \vdots \end{array}\\ \beta_{n} \end{array}\right]d=\left[\begin{array}{c} \begin{array}{c} d_{1}\\ d_{2\;}\\ \vdots \end{array}\\ d_{n} \end{array}\right]. \end{array}$$

#### 3.3.1. Weight Optimization by PSO

As we know that particle swarm optimization is an optimization technique [44], which can optimize a problem by repeatedly testing to enhance a candidate solution with relation to a given measure of quality [45]. Basically, the design process is based on the manner of birds, so that they can exchange the information by swarming behavior [46, 47].

Previously, we have suggested that by the help of PSO, the best position [48] can be estimated by improvement of the weights. So, weights must be optimized in case of PSO. Here, each particle has factors such as position vector *p*_*k*_ as well as velocity vector *w*_*k*_ [49, 50] and these [51] are expressed in

(14) $$\begin{array}{c} w_{k}^{n+1\;}=w_{k}^{n}+\beta \delta_{1}\left[g^{*}-p_{k}^{n}\right]+\gamma \delta_{2}\left[p_{k}^{*}-p_{k}^{n}\right], \end{array}$$

where *δ*_1_ and *δ*_2_ = random vectors between 0 and 1 [52].

 
*g*^*∗*^  = global best position
 
*β* and *γ* = learning parameters

In a typical PSO algorithm, if an inertia function *ɸ* (*n*) is used, *w*_*k*_^*n*^ has been replaced by *ɸ* (*n*) *w*_*k*_^*n*·*w*^ [53]. Now, this can be expressed as

(15) $$\begin{array}{c} w_{k}^{n+1\;}=\Phi w_{k}^{n}+\beta \delta_{1}\left[g^{*}-p_{k}^{n}\right]+\gamma \delta_{2}\left[p_{k}^{*}-p_{k}^{n}\right], \end{array}$$

where Φ € (0, 1).

Now, the weights are previously mentioned in Figure 2 as *w*= [*w*_*i*0_+ *w*_*i*1_*x*_1_+⋯⋯+*w*_*ij*_*x*_*j*_].

Furthermore, the weights are updated by using

(16) $$\begin{array}{c} w_{i}^{n+1}=\;\left(1-\gamma \right)w_{i}^{n}+\gamma g^{*}+\beta \delta_{n}. \end{array}$$

## 4. Result and Discussion

Here, we have used the BraTs 2020 dataset where it has used 278 MRI samples has been taken for both training and testing. In this work, 47 patient's data have been recorded in which 29 images for testing as well as 18 images for testing. All the exploratory analysis has been done with the python language with Google Co-lab in front end along with tensor flow tool in back end. Now, for the image segmentation by our planned method, IFRFCM has been presented in Figure 2.

Now for estimating the accomplishment of classification, we have taken one new technique that encompasses some additional things. It is purely based upon medical calculation and it is statistical software. Here, some new technical terms have been used and these are listed below:

For the diseased group, let

(17) $$\begin{array}{c} \text{Test Positive}=M,\\ \text{Test Negavtive}=N. \end{array}$$

For the nondiseased group, let

(18) $$\begin{array}{c} \text{Test Positive}=P,\\ \text{Test Negavtive}=Q. \end{array}$$

Disease prevalence: it is a statistical method which permits either the clinical experts or the researchers to estimate a person's chances of contracting a disease.

(19) $$\begin{array}{c} \text{Sensitivity}=\;\frac{M}{M+N},\\ \text{Specificity}=\frac{Q}{P+Q}. \end{array}$$

Positive predicted value (PPV): if the test case is positive, the probability for that particular disease is present and it is described as

(20) $$\begin{array}{c} PPV=\;\frac{\text{Sensitivity}\times \text{Prevalence}}{\text{Sensitivity}\times \text{Prevalence}+\left(1-\text{Specificity}\right)\times \left(1-\text{Prevalence}\right)}. \end{array}$$

Negative predicted value (NPV): if the test case is negative, the probability for that particular disease is not present and it is described as

(21) $$\begin{array}{c} \text{NPV}=\frac{\text{Specificity}\times \left(1-\text{Prevalence}\right)}{\left(1-\text{Sensitivity}\right)\times \text{Prevalence}+\text{Specificity}\times \left(1-\text{Prevalence}\right)}, \end{array}$$

(22) $$\begin{array}{c} \text{Accuracy}=\text{Sensitivity}\times \text{Prevalence}+\text{Specificity}\times \left(1-\text{Prevalence}\right). \end{array}$$

By the above descriptions and from the BraTs dataset, the accomplishments of various classification methods are estimated in Table 1.

From Figure 2, it has been monitored that the IFRFCM segmentation technique has the ability to detect the noisy image as well as the clear cancer region [54]. By the help of different parameters and number of iterations depicted in Figure 3, it has been observed that PSO-based ELM gives better classification accuracy as compared to the other classification models.

## 5. Conclusion

This research work has suggested 4 methods for the encephalon tumor detection process. Initially, the tumor region has been captured by MRI, all the images were divided, and the noisy images have been clearly found out by using the IFRFCM algorithm. After that, the features have been removed by the most commonly method, the GLCM method. Finally, the categorization or classification for finding out whether the tumor is cancerous or noncancerous has been investigated by the PSO-based ELM technique which gives an average classification accuracy rate of 99.47. Again, this proposed method can give better accomplishments if some deep characteristics have been applied.

## Figures and Tables

**Figure 1:** Workflow diagram of planned methodology.

**Figure 2:** Segmentation outcome. (a) Original image. (b) Noisy image. (c) IFRFCM outcome.

**Figure 3:** MSE of different techniques.

**Table 1:** Estimation of various classification accomplishments.

Techniques	Sensitivity	Specificity	PPV	NPV	Accuracy
PSO	0.91	0.84	96.23	93.35	95.61
SCA	0.93	0.86	96.38	93.42	98.01
ASCA	0.94	0.88	96.47	9351	98.32
ELM	0.97	0.91	97.82	94.73	98.88
PSO-based ELM	0.99	1.0	98.35	95.69	99.47

## Data Availability

The data will be available from the first author upon request.
